RETRACTED

# Apatinib Promotes Apoptosis of Pancreatic Cancer Cells through Downregulation of Hypoxia-Inducible Factor-1*α* and Increased Levels of Reactive Oxygen Species

**DOI:** 10.1155/2019/5152072

**Published:** 2019-02-04

**Authors:** Ke He, Lu Wu, Qianshan Ding, Farhan Haider, Honggang Yu, Haihe Wang, Guoan Xiang

**Affiliations:** ^1^Department of Biochemistry, Zhongshan School of Medicine, Sun Yat-sen University, Guangzhou 510080, China; ^2^Center for Stem Cell Biology and Tissue Engineering, Key Laboratory of Ministry of Education, Sun Yat-sen University, Guangzhou 510080, China; ^3^Department of General Surgery, Guangdong Second Provincial General Hospital, Guangzhou 510317, China; ^4^Department of Radiation and Medical Oncology, Zhongnan Hospital of Wuhan University, Wuhan University, Wuhan 430071, China; ^5^Department of Gastroenterology, Renmin Hospital of Wuhan University, Wuhan 430060, China; ^6^Department of Radiation and Medical Oncology, Hubei Key Laboratory of Tumor Biological Behaviors, Hubei Clinical Cancer Study Center, Zhongnan Hospital, Wuhan University, Wuhan, Hubei 430071, China

## Abstract

At present, apatinib is considered a new generation agent for the treatment of patients with gastric cancer. However, the effects of apatinib on pancreatic cancer have not been clarified. This study investigated the impact of apatinib on the biological function of pancreatic cancer cells and the potential mechanism involved in this process. Using the Cell Counting Kit-8 method, we confirmed that apatinib treatment inhibited cell proliferation *in vitro*. Moreover, the migration rate of pancreatic cells was inhibited. The effects of apatinib on apoptosis and cell cycle distribution of pancreatic carcinoma cells were detected by flow cytometry. The number of apoptotic cells was significantly increased, and the cell cycle was altered. Furthermore, we demonstrated that apatinib inhibited the expression of hypoxia-inducible factor-1*α* (HIF-1*α*), vascular endothelial growth factor, and markers of the phosphoinositide 3-kinase (PI3K)/Akt/mTOR signaling pathway, which increased the levels of reactive oxygen species *in vitro.* Apatinib significantly inhibited the biological function of pancreatic cancer cells. It promoted apoptosis, downregulated the expression of HIF-1*α*, and increased the levels of reactive oxygen species.

## 1. Introduction

Emphasized by the close relationship between disease incidence and mortality, pancreatic cancer is a highly fatal disease [1, 2]. Each year, >200,000 individuals die due to pancreatic cancer worldwide. In the USA, the 5-year survival rate of patients with pancreatic cancer is as low as 6% [3]. In most cases, patients with pancreatic cancer are asymptomatic until the disease reaches an advanced state, highlighting that this disease remains one of the most difficult to treat cancer [4]. Pancreatic cancer is not sensitive to radiotherapy or chemotherapy. Thus, an effective and safe treatment is urgently warranted. Over the past decade, it has been shown that the vascular endothelial growth factor (VEGF) and its homologous receptors, that is, the vascular endothelial growth factor receptors (VEGFR), play an important role in carcinogenesis [5–7]. Based on this evidence, therapeutic strategies against these targets (e.g., bevacizumab and panitumumab) have been widely studied. In addition, ziv-aflibercept and regorafenib were approved as second- and third-line treatment options, respectively [8].

RETRACTED

Apatinib—also termed YN968D1—is a novel oral antiangiogenic small molecule [9]. This agent selectively inhibits VEGFR-2, c-Kit, and c-SRC tyrosine kinases [10, 11]. Now in China, apatinib has been used for the treatment of gastric carcinoma patients [12, 13]. Considering the great patient population and lethality of pancreatic cancer in various countries, it is important to understand the pathobiology and signaling pathways involved in disease progression and develop novel therapeutic approaches. Agents such as aflibercept (a VEGF inhibitor) and axitinib (a VEGFR tyrosine kinase inhibitor) have been tested for the treatment of pancreatic cancers, with limited success [7]. However, the antitumor activity and potential molecular mechanism of apatinib against pancreatic cancer remain to be elucidated.

Activation of hypoxia-inducible factor-1 alpha (HIF-1 alpha) can affect the occurrence and development of pancreatic cancer. The expression of HIF-1*α* assists pancreatic cancer cells to adapt to hypoxia [14, 15]. In addition, it regulates the expression of downstream genes, such as VEGF. These effects increase the supply of blood to the pancreatic cancer lesions, leading to proliferation, angiogenesis, and metastasis [16]. Although the inhibitory effect of apatinib on VEGFR-2 has been determined, its impact on HIF-1*α* remains unknown.

In this study, the antitumor activities of apatinib on cell proliferation, cell cycle, migration, and apoptosis were analyzed *in vitro*. In addition, the expression of HIF-1*α* and alteration of the levels of reactive oxygen species (ROS) were assessed. Moreover, the expressions of markers of the PI3K/AKT/mTOR pathway—an important signaling pathway closely involved in the regulation of cell apoptosis—were detected [17]. We presented evidence that apatinib induced apoptosis in pancreatic cancer cells and exerts an effect on HIF-1*α* and ROS. These findings provide a novel molecular insight into the targets of apatinib.

RETRACTED

## 2. Materials and Methods

### 2.1. Antibodies and Reagents

The antibodies used in this study are as follows: GAPDH, HIF-1*α* rabbit mAb, bcl-2 rabbit mAb, caspase-3 rabbit mAb, Bax rabbit mAb, cleaved caspase-3 rabbit mAb, Akt rabbit mAb, phospho-Akt (Ser473) rabbit mAb, mTOR rabbit mAb, phospho-mTOR (Ser 2448) rabbit mAb, light chain 3B (LC3B) rabbit mAb, and goat secondary antibody to rabbit (horseradish peroxidase-conjugated). All antibodies were provided by Cell Signaling Technology (Cell Signaling, Boston, USA). Apatinib was purchased from Selleck (Houston, USA) and was dissolved in dimethyl sulfoxide. The final concentration of dimethyl sulfoxide in the treatment of the cells was controlled to <0.1% [18].

### 2.2. Cell Culture

The pancreatic cancer cell lines CFPAC-1 and SW1990 were obtained from the Cell Collection Center of Wuhan University (Wuhan, China). The cells were cultured in Iscove's Modified Dulbecco's Medium (IMDM; Gibco, New York, USA) containing 10% fetal bovine serum (FBS), at 37°C, with 5% CO_2_.

### 2.3. Cell Proliferation Assay

Twenty-four hours prior to treatment, CFPAC-1 and SW1990 cells were inoculated into 96-well plates. Subsequently, different drug concentrations (i.e., 0, 10, 20, 30, 40, and 50 *μ*M) in 10% FBS were used to treat these cells. In each well, 10 *μ*l Cell Counting Kit-8 (Beyotime, Shanghai, China) was mixed and the cells were cultured at 37°C for 1 h. The absorbance was measured using a microplate reader at 450 nm. All experiments were carried out in triplicate.

### 2.4. Migration and Wound Healing Assay

A cell migration assay was performed using the transwell chambers (8 *μ*M; Corning, New York, USA) [19]. We add the IMDM containing 10% FBS to the bottom of the chamber. Subsequently, CFPAC-1 and SW1990 cells (5 × 10^4^) in a serum-free IMDM, treated with different concentrations of apatinib, were mixed to the upper chamber of each well. Cells which adhered to the membrane were fixed using 4% paraformaldehyde and stained with 0.1% crystal violet dye. Migrated cells in the membrane were photographed from six different angles using an inverted microscope. The confluent monolayer cell plate was scraped using the tip of a 250 *μ*l pipette. Cells were cultured in the serum-free medium to measure the wound healing over a 48 h period.

### 2.5. Cell Cycle Analysis

After treatment with apatinib for 24 h, these cells were harvested and fixed using 75% ethanol overnight at −20°C. The following day, propidium iodide (PI) (50 *μ*g/ml) and RNase A (1 mg/ml) were added to the cell suspension for 0.5 h examined by flow cytometry (BD FACSCalibur, Becton Dickinson, San Jose, CA) and the proportions of cells in the G1, S, and G2 phases were analyzed [18].

RETRACTED

### 2.6. Analysis of Apoptosis

After reaching a confluence of 50-60%, the cells were treated with various concentrations of apatinib and harvested as previously described [18]. Subsequently, these cells were stained with annexin V-fluorescein isothiocyanate (FITC)/propidium iodide (PI), and the number of apoptotic cells was counted. These cells were analyzed by using the BD FACSCalibur in each experiment. All experiments were carried out in triplicate.

### 2.7. Reactive Oxygen Species Assay

After treatment with apatinib for 24 h, the cells were collected and incubated in 10 *μ*M 2′-7′dichlorofluorescin diacetate (DCFH-DA) (Beyotime, Shanghai, China) for 20 min at 37°C. Subsequently, the cells were washed and resuspended in a phosphate-buffered saline. The fluorescence intensity was determined using flow cytometry.

### 2.8. Western Blot Analysis

Briefly, CFPAC-1 and SW1990 cells were first collected using standard procedures. Total protein (40 *μ*g per sample) was then measured by the BCA Protein Assay Kit (Pierce Biotechnology, Rockford, IL), loaded for sodium dodecyl sulfate gel electrophoresis, and transferred onto polyvinylidene fluoride membranes (Millipore, Billerica, MA). The membranes were then blocked with skimmed milk at room temperature for 1 hour and incubated at 4°C overnight with primary antibodies against GAPDH, HIF-1*α*, Bax, bcl-2, caspase-3, cleaved caspase-3, Akt, phospho-Akt, mTOR, phospho-mTOR, and LC3B. Total levels of GAPDH were used as a control. Densitometric analysis was performed using the chemiluminescence imaging system (Alpha Innotech Corp., San Leandro, CA), and the relative protein expression was calculated after normalization of the target total protein.

### 2.9. Statistical Analysis

All experiments were performed in triplicate, and all results are expressed as means ± standard deviation (SD). The data were normally distributed, and the Student's *t*-test was used to analyze the statistical significance between experimental groups. When *P* < 0.05, the difference was considered to be statistically significant. Graphs were produced using GraphPad Prism 6 (La Jolla, CA). The SPSS V17 Student Edition Software was used for statistical analysis.

## 3. Results

### 3.1. Apatinib Inhibited Cell Proliferation in a Concentration- and Time-Dependent Manner

CFPAC-1 and SW1990 cells were treated with low-to-high concentrations (0-50 *μ*M) of apatinib to determine the cytological effect of apatinib on the proliferation of pancreatic cancer cells (Figure 1(a)). The IC_50_ for CFPAC-1 and SW1990 cells were 20.84 ± 1.62 *μ*M and 16.44 ± 1.48 *μ*M, respectively. Therefore, the 8 *μ*M and 16 *μ*M dosages of apatinib were used for further experimentation. Subsequently, we treated CFPAC-1 and SW1990 cells in an increasing time gradient, to further explore the capacity of apatinib to inhibit cell growth in a time-dependent manner. As shown in Figure 1(b), the inhibition of cell proliferation induced by treatment with apatinib increased in time-dependent manner. Collectively, apatinib inhibited the proliferation of pancreatic cancer cells in a concentration- and time-dependent manner.

RETRACTED

### 3.2. Apatinib Promoted Cell Cycle Arrest of Pancreatic Cancer Cells

Apatinib was used to treat pancreatic cells in a concentration-dependent manner. After 48 h, a relatively normal pattern of cell cycle was observed in untreated cells. CFPAC-1 and SW1990 cells were in the G1 phase (67.81 ± 2.93% and 67.34 ± 1.85%, respectively), while a lower proportion of cells was in the G2 phase peak (8.36 ± 3.41% and 6.36 ± 1.23%, respectively) and the S phase (23.83 ± 3.51% and 26.29 ± 1.34%, respectively). As shown in Figure 2, the cell cycle distribution of CFPAC-1 and SW1990 cells after treatment with 8 *μ*M apatinib was as follows: S phase (13.81 ± 1.56% and 13.69 ± 2.55%, respectively), G1 phase (80.55 ± 3.90% and 79.01 ± 3.15%, respectively), and G2 phase (5.62 ± 2.58% and 7.29 ± 1.46%, respectively). Following treatment with 16 *μ*M apatinib, these distributions were S phase (9.46 ± 0.91% and 10.67 ± 2.01%, respectively) and G1 phase (84.16 ± 3.54% and 85.13 ± 2.34%, respectively). The proportion of treated cells in the G1 phase was significantly increased, whereas that in the S phase was evidently reduced (*P* < 0.01). These results suggested that the effect of apatinib on cell cycle distribution was concentration-dependent, indicating that apatinib regulates pancreatic cancer cells at the G0–G1 phase in the process of karyomitosis.

### 3.3. Apatinib Inhibited Pancreatic Cell Migration

Furthermore, we examined the effects of apatinib on cell migration using the transwell assay. As shown in Figure 3(a), the migration effect was significantly reduced in cells treated with apatinib (*P* < 0.01). We found that apatinib significantly reduced cell migration in a concentration-dependent manner. The wound healing assay was performed to further validate the effect of apatinib on cell motility (Figure 3(b)). Consistent with the aforementioned experimental results, treatment with apatinib depressed the mobility of pancreatic cancer cells. Furthermore, the inhibition ratio increased in a concentration-dependent manner. These evidences suggested that apatinib may be a promising antitumor and antimetastatic drug.

RETRACTED

### 3.4. Apatinib Induced Apoptosis of Pancreatic Cancer Cells

Treatment with apatinib significantly increased the percentage of apoptotic cells in each cell (Figures 4(a) and 4(b)). In control cells, the percentages of apoptosis were 1.28 ± 0.30% and 9.21 ± 0.65%, respectively. In cells treated with 8 *μ*M apatinib, these values were 3.16 ± 0.89% and 21.46 ± 2.22%, respectively. In cells treated with 16 *μ*M apatinib, these values were 6.44 ± 0.88% and 30.02 ± 1.91%, respectively. Both dosages significantly increased the proportion of apoptotic cells (*P* < 0.05). Furthermore, protein levels of Bcl-2, Bax, and caspase-3 related to apoptosis were detected by western blotting. As shown in Figure 4(c), the expression of Bcl-2 was decreased after treatment of CFPAC-1 and SW1990 cells with 8 *μ*M apatinib, whereas those of Bax and cleaved caspase-3 were increased. These results suggested that apatinib promotes apoptosis in pancreatic cancer cells.

### 3.5. The Effects of Apatinib on the Generation of ROS

CFPAC-1 and SW1990 cells were treated with 8 *μ*M apatinib for 24 h prior to staining with DCFH-DA. The generation of ROS was estimated by measuring the fluorescence intensity of DCFH-DA. The fluorescence of CFPAC-1 and SW1990 cells treated with apatinib was significantly increased compared with that observed for control cells (Figure 5). These results demonstrated that the increased levels of ROS after treatment with apatinib promoted apoptosis of the pancreatic cancer cell.

### 3.6. Apatinib Inhibited the Expression of HIF-1*α* and Its Downstream Genes

Subsequently, we attempted to identify the potential molecular mechanism involved in the promotion of apoptosis by apatinib. Hence, we measured the expression of HIF-1*α*, VEGF, AKT, pho-AKT, mTOR, and phospho-mTOR through western blotting, after we treated pancreatic cancer cells with apatinib for 24 h. Compared with the control cells, treated pancreatic cancer cells presented a significant decrease in the expression of HIF-1*α* and VEGF (Figure 6(a)). As shown in Figure 6(b), the expression of total AKT protein kept unchanged under all experimental concentrations. However, killing with apatinib (8 *μ*M and 16 *μ*M) resulted in a significant decrease in the levels of phospho-AKT protein in each cell line. Concurrently, compared with those observed in control cells, the levels of phospho-mTOR protein of apatinib-treated pancreatic cancer cells were depressed. These findings suggested that cell apoptosis and growth inhibition induced by apatinib may be closely related to the downregulation of HIF-1*α* and VEGF. The downregulation of the AKT/mTOR pathway may also be partly involved in apoptosis. Moreover, the levels of light chain 3- (LC3-) II in apatinib-treated cells were found to be significantly higher than those reported in the control cells (Figure 6(b)). This increase in the level of LC3-II suggests the activation of autophagy after treatment of pancreatic cancer cells with apatinib.

RETRACTED

## 4. Discussion

Although pancreatic cancers are resistant to certain inhibitors of the VEGF pathway, we found that the proliferation and migration of pancreatic cancer cells were inhibited by apatinib in a concentration-dependent manner. In this study, we also showed that apatinib was cytotoxic to pancreatic cancer cells and the treatment induced apoptosis and loss of cell viability. Furthermore, we indicated that apatinib played a great inhibitory role in the migration of pancreatic carcinoma cells, in a concentration-dependent manner. This phenomenon was consistent with the clinical implications of apatinib, so as to be an effective option for further treatment in pancreatic cancer patients.

In China, apatinib is considered the new generation of oral antiangiogenesis drugs. Moreover, it is a potential third-line selection for the treatment of refractory gastric carcinoma [20]. Currently, clinical trials have been unable to provide definitive conclusions. However, in massively pretreated patients, the survival ratios including overall survival and progression-free survival were improved [21]. Angiogenesis refers to the formation of new blood vessels from previously existing vessels. Antiangiogenesis has been identified as an important treatment for several tumors, such as gastric and colon cancer.

Recently, a case report demonstrated a positive response to treatment with apatinib in a patient diagnosed with metastatic pancreatic cancer [22]. Moreover, another case report showed achievement of a progression-free survival > 11 months after administration of apatinib in a patient with pancreatic cancer-mediated malignant ascites [23]. It was popular in the therapy to incorporate antiangiogenesis factors with VEGF pathway inhibitors. Apatinib—a VEGFR-2 inhibitor—may inhibit endothelial cell migration and proliferation stimulated by VEGF, while simultaneously decreasing the tumor microvascular density. Therefore, it was approved as a promising VEGFR-2 inhibitor for the prevention of tumor-induced angiogenesis [24, 25].

Regarding the antitumor mechanism of apatinib, the currently available studies are mostly focused on antiangiogenesis [26, 27]. Interestingly, our work revealed that treatment with apatinib may inhibit the expression of HIF-1*α* and increase the levels of ROS. It has been reported that HIF-1*α* is highly expressed in pancreatic cancer tissues and cell lines, assisting tumor cells in adapting to hypoxic stress. Thus, HIF-1*α* plays a regulatory role in tumor angiogenesis and energy metabolism. In this study, we found that expressions of HIF-1*α* and its downstream gene VEGF were both significantly decreased in apatinib-treated cells versus those observed in control cells. In addition, we further discovered that the ROS levels of apatinib-treated cells were significantly higher than those reported in control cells. It was hypothesized that apatinib may inhibit the expression of HIF-1*α* in pancreatic cancer cells, thereby attenuating their ability to adapt to oxidative stress. Consequently, the levels of ROS were increased and eventually led to apoptosis. Another important factor promoting apoptosis in pancreatic cancer cells may be the inhibition of the AKT/mTOR signaling pathway. Our study showed that the expressions of p-AKT and p-mTOR in apatinib-treated cells were lower than those observed in control cells.

RETRACTED

Interestingly, we showed that in apatinib-treated cells the protein level of the autophagy marker LC3-II was elevated, whereas that of LC3-I was decreased. Previous studies have reported that the intracellular levels of ROS may lead to mitochondrial dysfunction, promoting autophagy [28]. This is consistent with the present results we observed *in vitro*. Autophagy has been recognized as an important catabolic process since the 1960s [29]. The key function of autophagy is to reduce the accumulation of toxic products or meet the change of energy requirement through recovering and redistributing cellular components [17, 30, 31]. It has been established that the Akt/mTOR signaling pathway is a significant regulator of apoptosis and autophagy [32]. The Ulk1 autophagic complex is negatively regulated by mTORC1 activation in the process of autophagy, consequently promoting autophagy and apoptosis [33, 34]. These results suggest that apatinib may be a potential candidate for the treatment of pancreatic cancer.

In summary, our present work revealed that apatinib plays a significant role in the biological function of pancreatic carcinoma cells. We provided new insight into the regulatory molecular mechanism of apatinib on apoptosis in pancreatic cancer cells. The results provide a promising new therapeutic option for pancreatic carcinoma patients. Nevertheless, further animal studies and clinical trials are warranted to confirm these findings. Moreover, research should focus on combinations of chemotherapy drugs.

## Figures and Tables

**Figure 1:** Apatinib inhibited cell proliferation in a concentration- and time-dependent manner. (a) Cell viability assays of CFPAC-1 and SW1990 cells treated with low-to-high concentrations of apatinib for 48 h. (b) The CFPAC-1 and SW1990 cells were treated with apatinib (8 *μ*M or 16 *μ*M) for different time intervals. The inhibitory activity was expressed as an inhibition rate. All experiments were performed in triplicate. The results represent mean ± standard deviation; *n* = 4, *P* < 0.05.

RETRACTED

**Figure 2:** Apatinib promoted cell cycle arrest in a concentration-dependent manner. The cell cycle distributions of the CFPAC-1 and SW1990 cells after treatment with apatinib (0, 8, and 16 *μ*M) for 24 h were determined through flow cytometry. All experiments were performed in triplicate.

**Figure 3:** Apatinib inhibited the migration of pancreatic cancer cells. (a) The migration of CFPAC-1 and SW1990 cells after treatment with apatinib (0, 8, and 16 *μ*M) for 30 h was assessed using the transwell assay. The migrated cells on the bottom surface of the filters were stained. (b) The movement ability of CFPAC-1 and SW1990 cells after treatment with apatinib (0, 8, and 16 *μ*M) for 48 h was detected using scratch wound healing assays. All experiments were performed in triplicate.

**Figure 4:** Apatinib induced apoptosis of pancreatic cancer cells. (a) Following the treatment of CFPAC-1 and SW1990 cells with various concentrations of apatinib (0, 8, and 16 *μ*M) for 24 h, these cells were stained using annexin V-FITC/PI and assessed by FACS analysis. (b) The quantitative analysis of the apoptotic cell numbers is shown. (c) The protein levels of Bcl-2, Bax, caspase-3, and cleaved caspase-3 are shown. All experiments were performed in triplicate. The bars represent mean ± standard deviation; ^∗^*P* < 0.05.

**Figure 5:** Apatinib induced apoptosis through an elevation of the levels of ROS. After treatment for 24 h, CFPAC-1 and SW1900 cells were stained using DCFH-DA. The fluorescence intensities of apatinib-treated and control cells are shown. All experiments were performed in triplicate. The bars represent mean ± standard deviation; ^∗^*P* < 0.05.

**Figure 6:** Apatinib inhibited the expression of HIF-1*α* and the AKT/mTOR pathway. (a) CFPAC-1 and SW1990 cells were treated with apatinib (0 or 16 *μ*M) for 24 h, and alterations in the expression of HIF-1*α* and VEGF were determined through western blotting. GAPDH was included as a loading control. (b) CFPAC-1 and SW1990 cells were treated with different concentrations of apatinib (0, 8, and 16 *μ*M) for 24 h, and the levels of phosphorylated AKT, mTOR, and LC3 were determined through western blotting. GAPDH was used as a loading control. All experiments were performed in triplicate.

## Data Availability

The data used to support the findings of this study are available from the corresponding author upon request.
